# Relative effectiveness and adverse effects of cervical manipulation, mobilisation and the activator instrument in patients with sub-acute non-specific neck pain: results from a stopped randomised trial

**DOI:** 10.1186/1746-1340-18-20

**Published:** 2010-07-09

**Authors:** Hugh Gemmell, Peter Miller

**Affiliations:** 1 Principal Lecturer Chiropractic Sciences, Department of Academic Affairs Anglo-European College of Chiropractic Bournemouth, Dorset, UK; 2 Senior Lecturer Chiropractic Sciences, Department of Academic Affairs Anglo-European College of Chiropractic Bournemouth, Dorset, UK

## Abstract

**Background:**

Neck pain of a mechanical nature is a common complaint seen by practitioners of manual medicine, who use a multitude of methods to treat the condition. It is not known, however, if any of these methods are superior in treatment effectiveness. This trial was stopped due to poor recruitment. The purposes of this report are (1) to describe the trial protocol, (2) to report on the data obtained from subjects who completed the study, (3) to discuss the problems we encountered in conducting this study.

**Methods:**

A pragmatic randomised clinical trial was undertaken. Patients who met eligibility criteria were randomised into three groups. One group was treated using specific segmental high velocity low amplitude manipulation (diversified), another by specific segmental mobilisation, and a third group by the Activator instrument. All three groups were also treated for any myofascial distortions and given appropriate exercises and advice. Participants were treated six times over a three-week period or until they reported being pain free. The primary outcome measure for the study was Patient Global Impression of Change (PGIC); secondary outcome measures included the Short-Form Health Survey (SF-36v_2_), the neck Bournemouth Questionnaire, and the numerical rating scale for pain intensity. Participants also kept a diary of any pain medication taken and noted any perceived adverse effects of treatment. Outcomes were measured at four points: end of treatment, and 3, 6, and 12 months thereafter.

**Results:**

Between January 2007 and March 2008, 123 patients were assessed for eligibility, of these 47 were considered eligible, of which 16 were allocated to manipulation, 16 to the Activator instrument and 15 to the mobilisation group. Comparison between the groups on the PGIC adjusted for baseline covariants did not show a significant difference for any of the endpoints. Within group analyses for change from baseline to the 12-month follow up for secondary outcomes were significant for all groups on the Bournemouth Questionnaire and for pain, while the mobilisation group had a significant improvement on the PCS and MCS subscales of the SF-36_v2_. Finally, there were no moderate, severe, or long-lasting adverse effects reported by any participant in any group.

**Conclusions:**

Although the small sample size must be taken into consideration, it appears that all three methods of treating mechanical neck pain had a long-term benefit for subacute neck pain, without moderate or serious adverse events associated with any of the treatment methods. There were difficulties in recruiting subjects to this trial. This pragmatic trial should be repeated with a larger sample size.

## Background

Neck pain is a common disorder [1-6]. About 70% of adults will experience neck pain during their lifetime, and its point prevalence in the general population is around 22% [1,5,7-12]. After low back pain, neck pain is the most common reason patients give for seeking chiropractic care, and the second most common reason for the use of spinal manipulation [13,14]. Treatment of neck pain is costly in terms of utilisation of health care services, disability, compensation payments and lost work productivity [3,4,15,16]. Manipulation and mobilisation are both commonly used by chiropractors, osteopaths and manipulative physiotherapists to treat neck pain [17-21]. Among chiropractors the Activator instrument is also a commonly used form of spinal manipulation [22-24].

The cause of neck pain is multifactorial and can be due to musculoskeletal conditions, trauma, systemic conditions, infections, inflammatory conditions or neoplasm [1,4]. Usually, the underlying cause of neck pain is non-specific and cannot be related to a particular pathology as a cause of the presenting symptoms [1,4,25].

Numerous systematic reviews [1-3,5,15,26,27] have assessed the evidence for the effectiveness of cervical spine manipulation and mobilisation in the treatment of non-specific neck pain. The results of these reviews for effectiveness are inconclusive with failure to show any one therapy as superior to any other. Five studies have directly compared cervical manipulation and mobilisation with inconclusive results [8-10,28,29]. The quality of these studies are, in the main, poor with inadequate sample sizes, inappropriate and non-validated outcome measures, inadequate follow-up and lack of a placebo comparison group.

Bogduk [30] suggests that for neck pain there are no data from any study determining the proportion of patients that are pain free after manual therapy. Moreover, Peloso and Gross [31] suggest that due to the uncertainty of the results obtained in the limited number of studies of manipulation and mobilisation for neck pain, further studies are needed to compare the different therapies available for neck pain.

Very few clinical trials have studied manual therapy for subacute neck pain [15,27,32,33], with the research emphasis being placed on those subjects with complaints lasting for longer than 6 months [34]. Further, there is a dearth of evidence for the long-term effects of treatments for subacute neck pain [35]. Evans et al. [36] also state that there is a paucity of research evaluating the efficacy of common treatments for acute and subacute neck pain and, therefore, there is a lack of evidence to determine if the treatment of subacute neck pain could reduce the occurrence of chronic neck pain. The category of subacute non-specific neck pain was selected for investigation to help fill the large gap in the literature regarding effective treatments for this category of neck pain.

Harm from cervical manipulation is unknown, but estimates range from one in 20,000 to five in 10,000,000 [2]. Ernst [37] states that manipulation of the cervical spine is associated with serious complications, and even minor adverse effects should be a contraindication to further spinal manipulation. However, this impression was based entirely on case reports. As part of the University of California Los Angeles (UCLA) neck pain study, adverse reactions to cervical manipulation and mobilisation were determined [7]. Over 30% of the participants had reactions to treatment. Increased neck pain and stiffness were the most common symptoms; however, there were 212 adverse symptoms reported from chiropractic care. Those randomised to manipulation were more likely than those randomised to mobilisation to report adverse effects within 24 hours of treatment. A recent paper in the physiotherapy literature suggests that the benefits of cervical manipulation have not been established, and the associated risks of manipulation could be very serious [19]. Di Fabio [38], based on a literature review, suggests mobilisation should be used as an alternative to cervical manipulation until more definitive information on the benefits and risks of manipulation are known. However, Cassidy et al. [39] in a recent study of stroke associated with GP visits and chiropractor visits found the risk was equal for patients consulting either practitioner. This suggests that cervical manipulation may not be a cause of stroke, but associated with a stroke in progress.

Due to difficulty in recruiting appropriate subjects to the study we stopped the trial. The purposes of the study were then to (1) describe the trial protocol, (2) report on the results obtained for relative effectiveness of the three types of manual therapy and their perceived adverse effects, (3) discuss the problems we encountered in conducting this study.

## Methods

We conducted a pragmatic, randomised comparative trial among patients with subacute (at least 4 weeks, but no longer than 12 weeks duration) non-specific neck pain. The study was conducted in the outpatient clinic of the Anglo-European College of Chiropractic (AECC) during two recruitment phases: January through July 2007 and January through March 2008. The study received ethics approval from AECC, and recruitment, assessments and data analyses were conducted at AECC.

### Participants

Participants were recruited through newspaper advertisements using the local newspaper and regional community magazines of the greater Bournemouth metropolitan area. All patients were examined by either of the two chiropractic clinicians involved in the study who made a clinical diagnosis of subacute non-specific neck pain. Inclusion criteria for the study were age 18-64 years; a new or recurrent episode of neck pain present for more than 4 weeks, but no longer than 12 weeks; neck pain that could extend to the shoulder region or upper extremities, and be accompanied by headache, but neck pain was more painful; the patient agreed not to take medication or receive other treatment for neck pain during the course of the study (paracetamol 500 mg 4 times a day was allowed as rescue medication); and a baseline pain level of at least 4 on the 11-point numerical rating scale. Exclusion criteria were treatment with any of the interventions during 6 months prior to recruitment to the study; specific neck pain due to fracture, neoplasm, infection, inflammatory arthropathy, radiculopathy or myelopathy; factors contraindicating manipulation, such as blood coagulation disorders, long-term use of corticosteroids, anticoagulant medications, history of neck surgery, stroke or transient ischaemic attacks; plans to relocate; inability to read or understand English; and third-party liability or workers' compensation claims.

### Randomisation

Randomisation was done on a block design using a computer-generated programme, http://www.randomization.com. Sequentially numbered sealed opaque envelopes were prepared by a researcher not involved with the study. During the trial the clinician opened the envelope marked with the next consecutive number and informed the patient about the treatment allocated. Participants and clinicians were not masked to the type of treatment.

### Study protocol

This was a pragmatic trial and all participants received oral reassurance about the usually benign course of non-specific neck pain; trigger point pressure release to active trigger points; postisometric relaxation stretching, exercise advice and ergonomic advice. Two experienced chiropractic clinicians delivered all study treatments. The first clinician is a registered chiropractor with 30 years of experience in general chiropractic practice. The second clinician is also a registered chiropractor with 15 years of experience in general chiropractic, and for the past six years has been lead tutor for adjustive technique. Both clinicians also have extensive experience in use of the Activator instrument and in mobilisation, as well as teaching these methods in an undergraduate chiropractic programme.

We asked participants to record their medication use, including all drugs taken for pain, in a specially designed diary during the first three weeks after beginning treatment. Participants were also asked to record perceived prevalence and time of onset and duration for each adverse effect in a diary during the first three weeks after starting treatment. The categories of adverse effects were similar to those used by Hurwitz et al. [7]: increased neck pain, stiffness and soreness; radiating pain and discomfort; tiredness/fatigue; headache; dizziness, imbalance; nausea, vomiting; blurred or impaired vision; ringing or noises in the ear; arm or leg weakness; arm or leg numbness; confusion, disorientation; depression, anxiety; and any other adverse effect. The diaries on medication use and adverse effects were collected by the clinician on the last treatment visit or the participant posted these in a stamped self-addressed envelope.

During the baseline visit, a clinician assessed the volunteer on the inclusion and exclusion criteria and informed the person about the study. A complete history of neck pain, associated conditions, red flags and prior treatment were recorded. Physical examination followed a standard format, including a neurological screen, looking for contraindications to manipulation and exclusions to participation. After this the clinician decided if radiographs were necessary. None of the participants required x-rays. Those who were eligible and agreed to participate were asked to read the Information Form and sign the Informed Consent Document. At this time the clinician gave the participant all the baseline demographic and outcome measures to complete. The clinician exited the room to allow the participant to complete the forms without interference.

### Interventions

The treating clinician determined the level and side of the manipulable lesions using his clinical judgement. Specific considerations were given to pain and movement restriction of individual spine segments from C1 to T4, localised tenderness and presence of paraspinal muscle tenderness and tautness. The same clinical assessment was used for all three groups. Participants in each group received, at no charge, two treatments per week for three weeks, and were treated until symptom free or had received the maximum of six treatments. The duration of a single treatment session was 10 to 15 minutes.

### Manipulation

Spinal manipulation is a passive and rapid movement of a joint beyond its active and passive limit of movement, but remaining within the limit of the joint's anatomical integrity. Participants received one to two dynamic thrusts, applied with high velocity low amplitude force, directed at one or more restricted upper thoracic or cervical spine segments. This approach to manipulation is commonly referred to as diversified technique.

### Mobilisation

Mobilisation involves repetitive low-grade passive movement with variation in amplitude. Participants received low velocity low amplitude movements applied to one or more restricted upper thoracic or cervical spine segments. The participant was supine and grade III posterior-anterior and transverse oscillations were applied to the articular pillar and spinous process.

The manner of delivery between manipulation and mobilisation differed, with mobilisation having rhythmically applied smaller movements within a joint's physiological range, whereas manipulation used a single impulse of high velocity and low amplitude beyond the physiological range of the joint.

### Activator Instrument

An Activator IV instrument was applied with the patient prone and with a setting of 1 for the Atlas and 2 for the cervical and upper thoracic segments. Participants received one thrust over the articular pillar in line with the facet joint of the restricted segment. The analytical procedure associated with Activator Methods was not used. The force delivered with this instrument was high velocity low amplitude within the physiological range of the joint.

### Outcome measures

All outcome measures were self-rated at entry and at the end of treatment by participants filling out all outcome measures while in the clinic, but without interference from the clinician. The outcome measures were also posted (with a stamped self-addressed return envelope) to the participants at 3, 6 and 12 months from the end of treatment.

Patient Global Impression of Change (PGIC) was the primary outcome measure [40] and is determined by self-assessment on a 7-point scale (1 = very much improved, 2 = much improved, 3 = minimally improved, 4 = no change, 5 = minimally worse, 6 = much worse, and 7 = very much worse). The PGIC is a single item extrapolated from the Clinician's Global Impression of Change (CGIC) tool [41]. It is used to assess response primarily in psychopharmacological research [42]. The CGIC assessment has been shown to be a valid outcome measure suitable for routine use, reliable, and it is sensitive to change [43]. The PGIC has been used as the primary outcome in trials of exercise and fibromyalgia [44], trials of the treatment of pain syndromes have adopted the PGIC as a primary outcome measure [45], and it has been suggested as useful in manual therapy research [42]. While change in mean group scores may be statistically significant, the change may be of little use to the clinician and patient [40,46-48]. Salaffi et al. [46] have determined that "much improved" or "very much improved" means a clinically important change for the patient. Therefore participants selecting one of these options were considered to have had a clinically meaningful improvement. The PGIC has been extensively used by pain researchers as a standard outcome and for comparison to other outcome measures [49-52]. It is commonly used to assess patient's own impressions of change [53,54]. It is intuitively logical when considering statistical significance and clinical significance [55]. Yalcin and Bump [56] assessed construct validity of the PGIC compared to three independent measures of improvement and they found appropriate and significant associations between the measures. Evangelou et al. [57] analysed 63 different treatments in 240 trials covering 18 conditions and found the PGIC assessments of the effects of treatment are on average similar to those of the CGIG with an OR = 0.98 (95% CI = 0.88 to 1.08). Farrar et al. [58] also found a high correlation between the CGIC and the PGIC, which they felt added credibility to the validity of the PGIC. They went on to use the PGIC as the "gold standard" to determine change in the numerical rating scale for pain that is clinically significant. Demyttenaere et al. [59] found patient rated global improvement was significantly associated with the Symptom Check List-90-Revised and the Beck Depression Inventory. They concluded that patients with major depressive disorder with at least moderate nonspecific pain consider improvement globally by using pain, depression, and anxiety in their overall impression of improvement. Demyttenaere et al. [59] feel this global judgement is more representative of the actually observed and clinically relevant status or change. Therefore, the primary endpoint with respect to relative effectiveness was the proportion of participants marking "much improved" or "very much improved" from baseline to the 12-month follow up. However, reliability in the form of internal consistency and test-retest reliability is difficult to determine for global impression of change scales as internal consistency relates individual items of a questionnaire to the total score (global scales are composed of a single question), and test-retest reliability would require subjects to rate global change twice for the same problem with the same period of improvement. Construct validity may be supported by looking at the relationship between physical outcomes and patient-reported outcomes [60].

A secondary outcome measure was the neck BQ developed by Bolton and Humphreys [25] for use in patients with non-specific neck pain. This self-assessment questionnaire contains separate pre- and post-treatment sections. It uses 11-point numerical rating scales for pain, functional and social activity, depression, anxiety, coping ability and fear avoidance behaviours. The instrument has been shown to be reliable, valid, responsive to change and able to detect and quantify clinically significant improvement [25,60-63]. All measurements were treated as continuous variables and analysed for differences between and within the groups using the total raw score. Other secondary measures included the Short-Form Health Survey (SF-36_v2_), and pain level taken from the neck BQ. SF-36_v2 _component subscales of physical health (PCS) and mental health (MCS) were treated as continuous variables and used to compare differences between and within the groups. This instrument is commonly used in research and has been shown to be reliable and valid [64-66]. The 11-point numerical rating scale for pain is a valid and reliable measure of pain intensity [67-70]. All measurements were treated as continuous variables and analysed for differences between and within the groups.

### Statistical analysis

There appeared to be some inequality at baseline so odds ratios between the groups for the PGIC were adjusted for the baseline covariants of age, gender, pain, quality of life, and disability using binomial logistic regression. Within group analyses from baseline to the 12-month endpoint for each of the secondary outcome measures were conducted using dependent t-tests. Differences between the groups for each of the secondary outcome measures for each of the follow up points were analysed by ANCOVA adjusted for the baseline covariants [71]. Intention to treat analysis was used, and the mean score for each group on each outcome was inputted for missing values. Statistical significance was set at P < 0.05. Statistical analyses were conducted by a researcher masked to group assignment and not involved in the conduct of the study using SPSS software version 16.0.

## Results

Between January 2007 and March 2008, 123 patients were assessed for eligibility. Reasons for exclusion of 76 patients were neck pain for longer than 12 weeks (n = 45), neck pain for longer than 12 weeks and pain <4 on the NRS (n = 12), pain <4 on the NRS (n = 7), cervical radiculopathy (n = 5), neck pain for less than 4 weeks (n = 2), contraindications to manipulation (n = 2), pain <4 on the NRS and nerve root lesion (n = 1), neck pain for longer than 12 weeks and headache worse than neck pain (n = 1), and spinal manipulation in prior six months (n = 1). In March of 2008 we had to terminate recruitment of patients. At that time 47 participants had been included. Of these 47 participants, 16 were allocated to manipulation, 16 to the Activator instrument, and 15 to the mobilisation group (figure 1).

**Figure 1:** **Flow chart for patient recruitment and follow up**. For each follow up point the number of participants completing each of the outcome measures is indicated.

Baseline data are shown in Table 1. The figure shows the number of participants who completed each of the outcomes at each of the four follow up periods (end of treatment, 3 months, 6 months and 12 months from the end of treatment). During the three-week treatment phase, three participants dropped out of the Activator instrument group, two from the mobilisation group, and one form the manipulation group. We were only able to ascertain the reason for withdrawal from treatment of one participant (manipulation group) and that was to care for a seriously ill spouse.

**Table 1:** Baseline variables of the three interventions (Activator, Manipulation and Mobilisation)

Variable	Activator	Manipulation	Mobilisation
Mean age (SD)	46.8 (11.8)	46.9 (9.1)	43.8 (13.0)

Mean BMI (SD)	25.6 (5.4)	27.6 (7.0)	24.7 (3.5)

Mean BQ raw score (SD)	30.2 (10.9)	32.2 (9.6)	25.6 (10.6)

Females %	81	69	87

Mean NRS for pain (SD)	6.7 (1.5)	6.0 (1.3)	4.9 (1.3)

Mean SF-36 PCS (SD)	40.6 (6.5)	45.3 (8.5)	44.5 (6.0)

Mean SF-36 MCS (SD)	49.2 (12.0)	47.2 (9.6)	48.0 (10.2)

### Primary outcome

Treatment was considered successful if the participant marked "improved" or "much improved" on the PGIC at the 12-month endpoint. In the Activator group 5 of 10 participants (50%) considered themselves to be improved, for the manipulation group this was 8 of 11 (73%), and for the mobilisation group 10 of 13 considered themselves improved (77%). Table 2 shows the adjusted odds ratios for the difference between groups on the PGIC. No significant differences were found between the groups for any of the follow up points.

**Table 2:** Comparison between treatment groups for Patient Global Impression of Change adjusted for baseline covariants

Time	Act v Man		Act v Mob		Man v Mob	
	OR	95% CI	OR	95% CI	OR	95% CI
**End**	0	0 to 0	0	0 to 0	1.2	0.78 to 19.58

**3**	1.4	0.13 to 17.56	2.6	0.06 to 112.81	5.8	0 to 0

**6**	1.5	0.13 to 17.56	13.8	0.63 to 299.67	2.8	0.06 to 122.80

**12**	3.8	0.39 to 37.18	3.3	0.27 to 40.61	1.2	0.09 to 15.96

End = end of treatment; 3 = 3 month follow up; 6 = 6 month follow up; 12 = 12 month follow up

OR = adjusted odds ratios

95% CI = 95% confidence interval

Act = Activator instrument, Man = manipulation, Mob = mobilisation

### Secondary outcomes

Comparisons between the groups on the neck BQ from baseline to each of the follow up points are shown in Table 3. There were no significant differences between the groups at any of the follow up points. All groups had a decrease in raw scores from baseline through to the 12-month follow up. Disability decreased by 13 points over 12 months in the Activator instrument group, 18 points in the manipulation group, and 15 points in the mobilisation group. A reduction of at least 13 points is considered a clinically significant improvement.

**Table 3:** Comparison between the treatment groups for the Bournemouth Questionnaire adjusted for baseline covariants

Time	Act v Man		Act v Mob		Man v Mob	
	Mean	95% CI	Mean	95% CI	Mean	95% CI
End	0.19	-10.63 to 11.03	-0.77	-14.42 to 12.95	-0.94	-13.56 to 11.69

3	1.57	-12.07 to 15.20	4.35	-15.68 to 24.38	2.78	-15.54 to 21.09

6	8.69	-4.46 to 21.83	8.57	-7.82 to 24.96	-0.86	-15.54 to 15.31

12	6.54	-9.03 to 22.10	5.68	-12.33 to 23.69	-0.86	-17.28 to 15.59

Mean = mean difference

End = end of treatment; 3 = 3 months; 6 = 6 months; 12 = 12 months

95% CI = 95% confidence interval

Act = Activator instrument, Man = manipulation, Mob = mobilisation

Table 4 shows the comparisons between the groups on neck pain from baseline to each of the follow up points. There were no significant differences between the groups at any of the follow up points. All groups had a decrease in pain from baseline to the 12-month follow up point. Pain decreased by 3 points in the Activator group, 4 points in the manipulation group, and 3 points in the mobilisation group. A reduction in pain of at least 2 points is considered a clinically meaningful improvement.

**Table 4:** Comparison between the treatment groups for pain adjusted for baseline covariants

Time	Act v Man		Act v Mob		Man v Mob	
	Mean	95% CI	Mean	95% CI	Mean	95% CI
End	0.81	-1.83 to 1.99	0.24	-2.19 to 2.62	0.13	-2.09 to 2.36

3	0.39	-1.58 to 2.35	1.33	-1.55 to 4.22	0.95	-1.69 to 3.58

6	1.96	-0.34 to 4.26	1.61	-1.26 to 4.48	-0.35	-3.05 to 2.35

12	1.72	-1.17 to 4.62	1.30	-2.05 to 4.65	-0.42	-3.47 to 2.63

Mean = mean difference

End = end of treatment; 3 = 3 months; 6 = 6 months; 12 = 12 months

95% CI = 95% confidence interval

Act = Activator instrument, Man = manipulation, Mob = mobilisation

Table 5 shows comparisons between the groups on the MCS subscale of the SF-36_v2 _from baseline to each follow up point. There were no significant differences between the groups at any of the follow up points. All groups had small improvements in the MCS from baseline to the 12-month end point. The Activator group had an improvement of 4 points, manipulation 3 points, and mobilisation 7 points.

**Table 5:** Comparison between the groups for the Mental Component Summary of the SF-36_v2 _adjusted for baseline covariants

Time	Act v Man		Act v Mob		Man v Mob	
	Mean	95% CI	Mean	95% CI	Mean	95% CI
End	-0.81	-8.75 to 7.14	5.81	-4.34 to 15.85	6.62	-2.66 to 15.89

3	-1.98	-10.57 to 6.61	-0.66	-13.28 to 11.96	1.32	-10.23 to 12.86

6	-1.28	-10.47 to 7.89	0.89	-10.55 to 12.34	2.18	-8.59 to 12.95

12	0.42	-7.74 to 8.59	-1.75	-11.19 to 7.69	-21.17	-10.78 to 6.44

Mean = mean difference

End = end of treatment; 3 = 3 months; 6 = 6 months; 12 = 12 months

95% CI = 95% confidence interval

Act = Activator instrument, Man = manipulation, Mob = mobilisation

Comparisons between the groups on the PCS subscale of the SF-36_v2 _from baseline to each follow up point are shown in table 6. There were no significant differences between the groups at any of the follow up points. All groups had small improvements in the PCS from baseline to the 12-month endpoint. The Activator group had an improvement of 2 points, manipulation 5 points, and mobilisation 8 points.

**Table 6:** Comparison between the groups for the Physical Component Summary of the SF-36_*v*2 _adjusted for baseline covariants

Time	Act v Man		Act v Mob		Man v Mob	
	Mean	95% CI	Mean	95% CI	Mean	95% CI
End	2.39	-3.79 to 8.57	1.67	-6.14 to 9.47	-0.73	-7.93 to 6.48

3	1.56	-4.01 to 7.12	-2.56	-10.73 to 5.61	-4.11	-11.59 to 3.36

6	-2.72	-10.04 to 4.59	-3.68	-12.81 to 5.46	-0.95	-9.55 to 7.64

12	-4.41	-12.48 to 3.66	-4.53	-13.87 to 4.80	-0.12	-8.64 to 8.39

Mean = mean difference

End = end of treatment; 3 = 3 months; 6 = 6 months; 12 = 12 months

95% CI = 95% confidence interval

Act = Activator instrument, Man = manipulation, Mob = mobilisation

### Adverse events

Fifteen subjects reported adverse events with manual therapy, seven with Activator, four with manipulation and four with mobilisation. All instances of side effects were minor and resolved within 1-3 days. Table 7 shows the type and number of adverse effects reported by each group.

**Table 7:** Adverse effects

Adverse symptom	Activator	Manipulation	Mobilisation
Mildly increased neck pain	7	4	2

Mild radiating pain	5	2	1

Mild arm weakness	1	0	0

Mild arm numbness	1	0	0

Mild headache	3	3	4

Mild fatigue	3	3	0

Mild dizziness	1	1	1

Mild muscle twitching	0	1	0

Values represent the number of subjects in each group experiencing the symptom. All symptoms were short-lived (1-3 days).

### Use of rescue medication

Ten subjects reported use of rescue medication, five with Activator, three with manipulation, and two with mobilisation (table 8).

**Table 8:** Number of participants in each group using rescue medication

Group	Rescue Medication	No Rescue Medication
**Activator**	5	8

**Manipulation**	3	12

**Mobilisation**	2	11

### Within group analysis

Table 9 shows the mean within group change from baseline to the 12-month endpoint. On the outcomes of the BQ and pain all groups had a significant improvement. The mobilisation group was the only group to show a significant improvement on the PCS and MCS subscales of the SF-36_v2_.

**Table 9:** Within group change from baseline to the 12-month end point

Outcome	Activator Mean (SD) 95% CI	Manipulation Mean (SD) 95% CI	Mobilisation Mean (SD) 95% CI
**BQ**	13 (12.3) 5.49 to 20.36*	18 (15.9) 8.27 to 28.57*	15 (13.9) 7.71 to 23.09*

**NRS**	3 (2.3) 1.93 to 4.69*	4 (2.7) 1.79 to 5.20*	3 (2.4) 1.60 to 4.27*

**PCS**	2 (4.8) -5.14 to 0.68	5 (8.5) -10.65 to 0.18	8 (6.2) -11.08 to -4.26*

**MCS**	4 (8.9) -9.79 to 1.04	3 (5.8) -6.53 to 0.88	7 (8.9) -11.62 to -1.74*

BQ = Bournemouth Questionnaire

NRS = numerical rating scale for pain

PCS = physical component summary of the SF-36_v2_

MCS = mental component summary of the SF-36_v2_

Mean = mean improvement

SD = standard deviation

* = significant at p < 0.05

## Discussion

The trial was not designed to evaluate the individual components of the treatments, but to compare the relative effect of adding a different form of spinal dysfunction correction to a package of care used by most chiropractors and osteopaths. This package of care consisting of TrP therapy, exercise advice and ergonomic advice may have its own beneficial effects [72-82], and we wanted to determine the benefit of adding each of the forms of manipulation used. We had difficulty in recruiting participants and stopped the trial before its expected completion.

### Key findings

On the primary outcome of patient global impression of improvement, there were no significant differences between the groups at any of the follow up points. For the secondary outcomes of disability (BQ) and pain based on improvement from baseline to the 12-month endpoint all groups had a statistically significant improvement. However, only the mobilisation group showed a statistically significant improvement from baseline to 12 months on quality of life measures (SF-36_v2_). This suggests that all groups exhibited long-term improvement without one being superior to the other. However, due to the small sample size the result could be explained by chance and must be interpreted with caution. Further research is necessary with larger sample sizes to determine if the result of equality between the groups is a true effect or simply due to chance.

If further studies also show that equal results may be achieved using either Activator, diversified or mobilisation, perhaps our understanding of the putative lesion we treat may need to be revised. Currently, most osteopaths and chiropractors would suggest that manipulation restores normal joint play to a dysfunctional spine joint [83-91]. We now know that the surrounding fascia of a spine joint contains many more sensory receptors than the spine joint itself [87-91]. Recent research suggests that mechanical stimulation of an acupuncture needle and manual therapy procedures affect the network of fibroblasts via a process called mechanotransduction that can affect gene expression within the cell explaining the long-term effects achieved with these therapies [91-96]. This would also help explain how different methods of mobilisation from reflex methods to HVLA manipulation seem to have equal effects [5,10,15,26,27,29,97].

### Adverse effects

A recent large cohort study [98] did not find any severe adverse effects from chiropractic manipulation. The only symptoms perceived by participants in the current study as being adverse were minor and short-lived. Surprisingly the Activator instrument group had a higher proportion of these adverse effects as compared to manipulation, and mobilisation had a higher proportion of adverse effects as compared to manipulation. The reason why the Activator instrument was perceived by participants as being possibly harmful may be due to the fact we did not go into great detail about each treatment, but gave enough information for the participant to make an informed decision about participating. Further, the instrument has a mechanical, surgical appearance and the 'clicking' noise may have added to this concern. Also, patients' naïve to chiropractic care were enrolled in the study. Therefore, it is possible a nocebo effect could have occurred.

We have no explanation as to why mobilisation was perceived as more likely to cause an adverse effect compared to manipulation other than to suggest that while manipulation involved a quick thrust, segmental mobilisation was delivered to a specific point and mobilised over a longer period of time. If the point being mobilised was tender, then the participant may have viewed this as harmful.

A greater proportion of those in the Activator instrument group had to resort to rescue medication as compared to those in the manipulation and mobilisation groups. This may be explained by a significantly higher level of pain in the Activator instrument group at baseline.

### Difficulties in recruitment

The major problem we had with recruitment was overestimating the effect of advertising and the lack of adequate time for screening and treating patients in the study. We limited advertising to the major newspaper and magazines of the Bournemouth metropolitan area. Perhaps increasing coverage to radio and billboards would have helped in recruitment. Initially advertising was so successful that we had a waiting list of patients to be screened and we did not have enough time allocated to see the patients. Due to the stringent eligibility criteria, particularly the necessity for the subject to have sub-acute neck pain, by the time we were able to see the patient he/she was no longer able to meet the eligibility criteria. Both clinicians teach full-time on the undergraduate and postgraduate programmes and when we were able to devote more time to this study the advertising was not drawing the numbers as it had done initially. The Bournemouth area has a catchment of about 300,000 people and this may have been a limiting factor as compared to a large metropolitan area such as London. We then reached a point where we were no longer able to advertise further, due to a lack of funds, and had to stop the trial.

Our problems with recruitment were similar to those noted by Vernon et al. [99] in their study of tension-type headache. We considered a multicentre study may be a way in the future to obtain larger sample sizes; however, Vernon et al. [99] noted a problem with this approach in that it produced variation in delivery of trial protocols. Perhaps if this factor can be controlled a multicentre study could be a way of increasing numbers in a trial.

While we gave free care to all participants to increase participation, perhaps remuneration for participating could have increased the number of those willing to be involved. However, this would affect external validity of the study as those being paid to participate may be fundamentally different to those who pay for their care.

Upon reflection we feel a dedicated research centre with full-time practitioner-researchers would be one way of solving the perennial problem of recruitment, assuming grants are available for such a venture. This would be particularly appropriate for studying the relative effectiveness of the various therapeutic interventions used in manual therapy and would allow generalisability to standard chiropractic and osteopathic care.

### Comparison with other studies

Our finding of mobilisation causing more adverse effects than manipulation is in contrast to the study of neck pain by Hurwitz et al. [7] in which mobilisation was shown to have fewer adverse effects. As mentioned above, this could be due to the nocebo effect in participants' naïve to the different methods of chiropractic treatment. It is difficult to directly compare our study to this study as we included subacute neck pain patients while the study by Hurwtiz et al. included both subacute and chronic neck pain patients. Similar to the study by Hurwitz et al. we found the most commonly occurring adverse effect to be neck pain, stiffness/soreness. In our study 27% of those in the manipulation group had this symptom (28% in the Hurwitz et al. study), and 15% in the mobilisation group had this symptom (22% in the Hurwitz et al. study). In comparison 54% of those in the Activator instrument group had the same adverse symptom.

Previous randomised clinical trials have directly compared manipulation, mobilisation and the Activator instrument [96]; however, only one previous study has assessed the long-term effectiveness of manipulation versus mobilisation [10]. An evaluation of the effect of manual therapies on neck pain was investigated by Dziedzic et al [100], and they found no additional effect after six months when adding manipulation to exercise and advice. This is different to our study where we found a significant difference from baseline to 12 months within all groups.

To our knowledge, this present study is the first randomised clinical trial to compare the long-term effectiveness of manipulation, mobilisation and the Activator instrument for subacute non-specific neck pain. Our results agree with the study of Hurwitz et al. in that manipulation and mobilisation basically give comparable clinical results. One difference in the studies is that the study by Hurwitz et al. had a 6-month follow up while we had a 12-month follow-up.

### Limitations

Our study has several limitations. Firstly, the participants could not be masked to treatment, and neither were the clinicians masked to group assignment. We tried to avoid bias by having all outcome measures self-assessment instruments that participants did not complete in front of the clinicians. Secondly, by not having a placebo control group the results obtained may be explained by non-specific effects due to the attention given to the participants in each of the groups. Further, it is possible that the clinical improvement observed could be due to the myofascial therapy that all subjects received and the manipulative therapies were irrelevant to the outcome. Thirdly, we cannot exclude the possibility that patients with specific causes of neck pain may have participated in the study. However, we feel this is unlikely as we required a firm diagnosis of non-specific neck pain, followed by strict inclusion criteria. Those with specific causes of neck pain are unlikely to change the results of the study, as we would expect that they were equally distributed over the three arms. Finally, the disproportionate dropout rate for the Activator group compared to the other groups could also be a limitation of the study.

As we had to end recruitment early, we conducted a power analysis post hoc. Based on the PGIC comparing the Activator instrument group and the manipulation group, the PS programme version 2.1.31 http://biostat.mc.vanderbilt.edu/ was used to calculate power achieved. At a power of 0.80 and alpha of 0.05, 18 subjects per group were needed. The limited sample size we had gave us a power of 0.75. Therefore, the study was underpowered and subject to Type II error. Due to this limitation, the study has to be considered a pilot study.

The pragmatic design of this study we feel helps in external validity. None of the eligible patients refused to participate, we had few drop-outs, we used manipulative techniques commonly used in chiropractic practice, and had the participants engage in exercises, gave them myofascial therapy and clinical advice allowing generalisability to most modern chiropractic practices. However, the study was underpowered making it difficult to be generalised. Further factors affecting generalisability were our stringent inclusion criteria and the fact all subjects were recruited through advertising in local newspapers. These volunteers also received care free of charge. It is possible that such volunteers, receiving care for free are not the same as patients who generally seek chiropractic or osteopathic care.

## Conclusion

Our trial was stopped early due to an inability to recruit participants. However, our limited sample suggested a significant long-term improvement in subacute non-specific neck pain for all groups. Based on the comparable outcomes and low risk of adverse effects, chiropractors and osteopaths may obtain equally effective results by treating neck pain patients with manipulation, the Activator instrument, or mobilisation. However, the result must be treated with caution due to the small sample size and, this interesting finding needs to be confirmed in larger trials.

## Competing interests

The authors declare they have no non-financial competing interests. A portion of the study was funded by the National Institute of Chiropractic Research, USA a subsidiary of Activator Methods.

## Authors' contributions

HG conceived and designed the study, HG and PM acted as clinicians and project managers for the study. HG wrote the first draft of the manuscript, and both authors read and approved the final draft.
